The article "Serological and Entomological Study of Dengue in Dang and Chitwan Districts of Nepal" was retracted in 2022. Reason: lack of ethics approval or compliance.

# Serological and Entomological Study of Dengue in Dang and Chitwan Districts of Nepal

**DOI:** 10.1371/journal.pone.0147953

**Published:** 2016-02-01

**Authors:** Rojina Shrestha, Narayan Dutt Pant, Ganga GC, Srinivas Thapa, Biswas Neupane, Yogendra Shah, Ishan Gautam, Basu Dev Pandey

**Affiliations:** 1 Department of Microbiology, Trichandra multiple campus, Kathmandu, Nepal; 2 Department of Microbiology, Grande International Hospital, Dhapasi, Kathmandu, Nepal; 3 Everest International Clinic and Research Center, Kathmandu, Nepal; 4 Institute of Science and Technology, Tribhuvan University, Natural History Museum, Kathmandu, Nepal; Metabiota, UNITED STATES

## Abstract

A descriptive cross-sectional study was carried out among 264 suspected dengue patients in two districts (Dang and Chitwan) of Nepal from June 2013 to November 2013. The anti-dengue IgM positivity was found to be (51/264)19.31% by capture ELISA, of which 21 (41.2%) were male and 30 (58.8%) were female. Symptoms of seropositive cases were fever, anorexia, nausea, headache, retro-orbital pain, skin rashes, and myalgia. Hematological features like thrombocytopenia and leucopenia were found to be significantly associated with the dengue fever (DF). Discarded tires were found as the commonest breeding habitats for the dengue vectors. Higher sero-positivity was recorded from the area having higher Breteau index (BI). The pH, chloride ion concentration and the salinity of the water from breeding habitats were found to be ranging from 6.9±0.82 to 8, 103.33±17.52 mg/L to 140.65 mg/L, and 0.19±0.032 ppt to 0.25 ppt respectively. This study may be helpful for the health authorities and public health workers for early diagnosis of DF and for the improved preventive measures to be adopted in the epidemic and possible epidemic areas.

## Introduction

Dengue is a mosquito-borne viral infection endemic to most tropical and subtropical regions around the world, predominantly in urban and sub-urban areas [1, 2]. It is caused by four antigenically distinct serotypes of dengue virus (DENV 1–4) belonging to the family *Flaviviridae* and genus *Flavivirus*. Dengue viruses are transmitted to human by *Aedes aegypti* and *Aedes albopictus*. The infection is responsible for causing a spectrum of illness ranging from asymptomatic or mild febrile illness, dengue fever (DF), to severe and fatal hemorrhagic diseases, dengue hemorrhagic fever (DHF) and dengue shock syndrome (DSS) [3].

Infection with one serotype provides homologous long-lasting immunity to the same serotype but infection with heterologous serotypeslead to severe form of dengue that is DHF and DSS [4, 5].

Dengue fever is characterized by febrile illness with severe headache, retro-orbital pain, myalgia or arthralgia, nausea or vomiting, skin rashes while DHF is characterized by high fever lasting for 2 to 7 days, hemorrhagic symptoms (induced by leakage of plasma), thrombocytopenia and circulatory failure in severe cases. The condition of some patients progresses to shock due to severe plasma leakage, known as DSS leading to death.

The article "Serological and Entomological Study of Dengue in Dang and Chitwan Districts of Nepal" was retracted in 2022. Reason: lack of ethics approval or compliance.

The grading system of dengue fever has been established based on clinical and laboratory findings. Theoretically, DF should be relatively benign disease, while DHF might be potentially life threatening [6, 7]. The global prevalence of dengue cases is increasing dramatically in recent decades. It is estimated that over 2.5 billion people live at high risk of getting dengue infection with an incidence of 50–100 million cases and several thousands of deaths annually [8]. The disease is endemic in Africa, Latin America, Eastern Mediterranean, Western Pacific and South East Asia. Around 1.8 billion people residing in South East Asia and the Western Pacific region are at risk of dengue. During the past decade, the numbers of DENV infections increased in South Asia and DF/DHF epidemics occurred in Bhutan, India, Maldives, Bangladesh and Pakistan [6, 9]. Nepal is at higher risk of the introduction and establishment of DENV as the country is open bordered (where there is no restriction in travel and trade across the borders) by India and there is high frequencies of travel and trade across the borders.

The first case of dengue in Nepal was recorded in a foreigner in Chitwan in 2004 and subsequently the larger outbreak occurred in 9 districts of Terai region in 2006 with 23 confirmed dengue cases following the Indian epidemic of DF/DHF in September-October 2006 [6, 10, 11]. After four years another significant outbreak occurred in 2010 in Chitwan with at least 359 confirmed dengue cases [12]. From the observations above it can be concluded that dengue is a significant problem in the districts of Terai region of Nepal including Chitwan and Dang.

In Nepal there is lack of proper diagnostic facilities. Due to which the diagnosis of dengue cases is based solely on the patient’s clinical symptoms [10]. Nepal has no dengue surveillance programs targeting infections of dengue virus through the reports of clinicians [13]. Despite the geographical expansion and significantly high morbidity and mortality caused by infection of dengue virus in Nepal, very limited information on the distribution and abundance of mosquito vectors for dengue virus is available. A few entomological studies conducted in Nepal have revealed the presence of the dengue vectors (*Aedes aegypti* and *Aedes albopictus*) in some parts of Nepal ranging from Terai lowlands and Siwalik hills to Middle Mountain regions. They are commonly present up to 1350 m in Kathmandu and rarely up to 1750 m to 2100 m in Dhunche, Rasuwa district of Nepal [14].

The article "Serological and Entomological Study of Dengue in Dang and Chitwan Districts of Nepal" was retracted in 2022. Reason: lack of ethics approval or compliance.

In this study, clinical and laboratory-based surveillance systems were initiated in Dang and Chitwan districts. Additional medical entomology surveys were performed with emphasis on the abundance of breeding sites.

## Methods

### Statement regarding ethical approval

Patient’s consent form was used to obtain written informed consent from patients or the patient’s guardians (in case of minors). The ethical committee of Trichandra multiple campus, Kathmandu, Nepal approved the consent procedures as well as the study. The field studies did not involve endangered or protected species. In case of the study carried out in private land, the permission was obtained from the owner of the land. Since the area was not a protected area, for the study conducted in public area no permission was required.

A descriptive cross-sectional study was carried out in Dang (latitude 28°N and longitude 82°E) and Chitwan (latitude 27°N and longitude 84°E) districts of Nepal from June 2013 to November 2013. The total 264 (130 from male and 134 from female) serum samples were collected from patients (out patients) attending Bharatpur Hospital, Chitwan, Rapti zonal hospital, Dang and Rapti sub-regional Hospital, Dang. Only the patients with chief complain of febrile illness with two or more symptoms like ocular pain, headache, rash and arthralgia or myalgiawere included in the study. Out of 264 serum samples, 125 serum samples were collected from Bharatpur Hospital, Chitwan, 75 serum samples from Rapti Zonal Hospital, Dang and 64 serum samples from Rapti Sub-Regional Hospital, Dang. As suggested by inclusion and exclusion criteria specified by WHO, a case was excluded if routine tests suggested bacterial or any other diseases [6]. Common symptoms, duration of illness, travel history, occupation, related symptoms in other family members, address, age and sex of the patients were recorded through questionnaires. The hematological tests were done at the respective hospitals attended by the patients. Serum samples were transported to Everest International Clinic and Research Center, Kathmandu, by maintaining reverse cold chain and anti-dengue IgM was detected by Human Dengue IgM capture ELISA (Human GeseellschaftfÜr biochemical and diagnostic mbH, Germany). The entomological study was conducted in Dang and Chitwan. The potential habitats of *Aedes* mosquitoes were searched throughout the residential areas for the presence of immature dengue vectors. To precisely estimate the sizes of locally established vector populations, larvae and pupae were collected. The technique used for the collection was dropper and dipper method. The larvae and pupae were transported in plastic cups to the Natural History Museum, Kathmandu and reared by placing in different vials for emergence of adult mosquitoes [15]. The mosquitoes were identified on the basis of different morphological characters by using taxonomic keys published by Darsie and Pradhan [16]. Both of the dengue vectors (*Aedes aegypti* and *Aedes albopictus*) were found to be present in Chitwan and Dang. One hundred and sixty wet containers containing larvae and pupae of dengue vectors were examined which were categorized into eight different container types; discarded tires, plastic buckets, metal drums, roofs, cemented tanks, plastic tanks, plastic bottles and earthen pots. The physiochemical parameters (pH and salinity) of the water of the breeding habitats of vectors were determined following WHO guideline [17]. The pH of the water was determined by using pH meter while salinity of the water was determined by calculating the chloride ion concentration by Mohr’s method. Based on data collected district wise, *Aedes* index (AI), Container index (CI), Breteau index (BI) and breeding preference ratio (BPR) of dengue vectors for different containers were calculated.

The article "Serological and Entomological Study of Dengue in Dang and Chitwan Districts of Nepal" was retracted in 2022. Reason: lack of ethics approval or compliance.

### Statistical analysis

Data were analyzed using SPSS version 16.0. Values were expressed as mean ± standard deviation (SD). Crude odds ratio (OR) and 95% confidence intervals (CI) were calculated. Chi-square test was applied and the value of significance for all statistical tests was p value < 0.05.

Procedures of the study follow the compliance and regulations.

## Results

### Serological test

Serologically, 51(19.31%) serum samples out of 264 samples were found to be confirmed positive for anti-dengue IgM antibody. The ratio of the male to female participants was 1:1.03.

Among the seropositive dengue cases, 21 (41.2%) cases were male and 30 (58.8%) were female. Statistically, there was no significant difference between genders and positive serological results.

To find out the age wise distribution of seropositive dengue cases the study subjects were grouped with different intervals in terms of age. Seroprevalence rate of the age group less than 15 years old was 17.64% (12/68). Similarly, seroprevalence rate of the age group 15–50 years old was found to be 19.59% (29/148) and that of the age group more than 50 years old was 20.83% (10/48). Statistically, there was no significant difference between the age and the disease occurrence (Table 1).

**Table 1:** Age wise distribution of seropositive dengue cases.

Age	Total no. of samples	No. of positive samples (%)
<15 years	68	12 (17.64)
15–50 years	148	29 (19.59)
>50 years	48	10 (20.83)

Among the 51 seropositive dengue cases, Bharatpur Hospital(BH), Chitwan, accounted for 47 (92.156%) cases, Rapti Zonal Hospital(RZH), Dang accounted for 3 (5.882%) and Rapti Sub-regional Hospital(RSH), Dang accounted for 1(1.96%) of the cases (Fig 1). There was significant difference in anti-dengue IgM seropositivity in the patients from hospital in Chitwan and those from hospitals in Dang (p<0.05).

The article "Serological and Entomological Study of Dengue in Dang and Chitwan Districts of Nepal" was retracted in 2022. Reason: lack of ethics approval or compliance.

**Fig 1:** Hospital wise distribution of seropositive cases.

Among the dengue seropositive cases, the common clinical features were anorexia (60.78%) with an odds ratio of 7.7 (3.65–16.25), headache (78%) with an odds ratio of 2.19 (1.06–4.51), myalgia (75%) with an odds ratio of 1.3 (0.64–2.57), nausea (58.82%) with an odds ratio of 2.92 (1.56–5.46), retro-orbital pain (17.6%) with an odds ratio of 2.83 (1.16–6.89), abdominal pain (15.69%) with an odds ratio of 0.74 (0.32–1.68) and skin rashes (9.8%) with an odds ratio of 3.2 (0.97–10.53) (Table 2) but no signs of hemorrhage were seen.

**Table 2:** Clinical features of seropositive and seronegative cases.

Symptoms	ELISA positive cases (n = 51)	ELISA negative cases (n = 213)	Odds ratio (95% CI)	p-value
Headache	**40(78.43%)**	**133(62.4%)**	**2.19 (1.1–4.5)**	**0.018**
Anorexia	**31(60.78%)**	**75(35.21%)**	**7.7 (3.7–16.3)**	**0.01**
Nausea	**30(58.82%)**	**71(33.33%)**	**2.92(2–5.5)**	**0.01**
Myalgia	**38(74.5%)**	**148(69.48%)**	**1.3 (0.6–2.6)**	**0.49**
Retro-orbital pain	**9(17.6%)**	**15(7.04%)**	**2.83 (1.2–6.9)**	**0.018**
Skin rash	**5(9.8%)**	**7(3.29%)**	**3.2(1–10.5)**	**0.045**
Abdominal pain	**8(15.69%)**	**43(20.19%)**	**0.74(0.3–1.7)**	**0.47**

Out of 51 dengue seropositive cases, thrombocytopenia was seen in 31 (60.78%) cases and leucopenia in 38 (75%) cases. Increased hematocrit level was found in 6 (11.76%) cases (Table 3). The mean leukocyte count was 7279 ± 1170 / mm^3^ while the mean thrombocyte count was 109000 ± 51739 / mm^3^. The mean hematocrit level was 36.12±9.6%. Thrombocytopenia (p<0.05) and leucopenia (p<0.05) were found significant whereas increased hematocrit level was not found significant in dengue seropositive cases.

**Table 3:** Hematological features of seropositive cases.

Laboratory features	Positive cases	p- value
Leucopenia	**38 (75%)**	**0.014**
Thrombocytopenia	**31 (60.78%)**	**0.011**
Increased hematocrit	**6 (11.76%)**	**0.133**

### Entomological survey

Eight different containers were searched for the immature dengue vectors. Discarded tires were found with the highest BPR of 1.15 and 1.14 in both Chitwan and Dang respectively, and there was statistical significance (p<0.05) (Tables 4 and 5).

The article "Serological and Entomological Study of Dengue in Dang and Chitwan Districts of Nepal" was retracted in 2022. Reason: lack of ethics approval or compliance.

**Table 4:** Breeding preference ratio of the vector larvae of Chitwan district.

Breedingsite	Numbers of containers with water	Percentage of containers with water (X%)	Numbers of containers with larvae or pupae	Percentage of containers with larvae or pupae (Y%)	BPR (Y/X)
Discarded tires	**65**	**68.4**	**46**	**79.31**	**1.15**
Plastic buckets	**6**	**6.31**	**2**	**3.44**	**0.54**
Metal drums	**2**	**2.1**	**1**	**1.72**	**0.81**
Earthen pots	**5**	**5.3**	**3**	**5.17**	**0.98**
Roofs	**2**	**2.1**	**1**	**1.72**	**0.81**
Cemented tanks	**5**	**5.3**	**0**	**0**	**0**
Plastic tanks	**4**	**4.2**	**2**	**3.44**	**0.81**
Plastic bottles	**6**	**6.3**	**2**	**3.44**	**0.54**
Total	**95**	**100**	**58**	**100**	

**Table 5:** Breeding preference ratio of the vector larvae of Dang district.

Breeding site	Numbers of containers with water	Percentage of containers with water (X%)	Numbers of containers with larvae or pupae	Percentage of containers with larvae or pupae(Y%)	BPR (Y/X)
Discarded tires	**36**	**55.38**	**19**	**63.33**	**1.14**
Plastic buckets	**2**	**3.07**	**1**	**3.33**	**1.08**
Metal drums	**3**	**4.61**	**0**	**0**	**0**
Earthen pots	**5**	**7.69**	**2**	**6.66**	**0.86**
Roofs	**2**	**3.07**	**1**	**3.33**	**1.08**
Cemented tanks	**9**	**13.84**	**5**	**16.66**	**1.2**
Plastic tanks	**4**	**6.15**	**2**	**6.66**	**1.08**
Plastic bottles	**4**	**6.15**	**0**	**0**	**0**
Total	**65**	**100**	**30**	**100**	

*Aedes* index (AI), Container index (CI), and Breteau index (BI) of Chitwan were found to be 21.1%, 61.05% and 61.05%, respectively. AI, CI and BI of Dang were 17.1%, 46.15% and 31.25%, respectively. BI in Chitwan was found to be significantly higher in comparison to that in Dang (p<0.05). Statistically, there was no significant difference between AI and CI of Chitwan and those of Dang.

In this study, the physiochemical characteristics (pH, chloride ions concentration and salinity) of the water of the habitats of *Aedes* mosquito were determined (Table 6). The result showed that the *Aedes* larva could survive within the range of pH6.9±0.82 to 8. The chloride ion concentration was (140.65 mg/L) in metal drums followed by discarded tires (119.4± 34.37mg/L), earthen pots (117.46±56.01 mg/L), cemented tanks (116.01± 23.05 mg/L), plastic tanks (105.86±35.9 mg/L) and plastic buckets (103.33±17.52 mg/L). The salinity of the water was found to be (0.25±0.00 ppt) in the metal drums followed by earthen pots (0.21±0.101 ppt), discarded tires (0.21±0.062 ppt), cemented tanks (0.21± 0.041), plastic tanks (0.19±0.065 ppt) and plastic buckets (0.19±0.032 ppt). This result showed that the mosquitoes can breed in the water with chloride ion concentration ranging from 103.33±17.52 mg/L to 140.65 mg/L and salinity ranging from 0.19±0.032 ppt to 0.25±0.00 ppt.

The article "Serological and Entomological Study of Dengue in Dang and Chitwan Districts of Nepal" was retracted in 2022. Reason: lack of ethics approval or compliance.

**Table 6:** Physiochemical characteristic of water of breeding habitats of *Aedes* mosquito.

Habitats	Physiochemical Parameters		
	pH(Mean ± SD)	Chloride ions concentration(mg/L) (Mean ± SD)	Salinity (ppt)(Mean ± SD)
Discarded tires (n = 42)	**7.6 ± 0.75**	**119.4 ± 34.37**	**0.21 ± 0.062**
Cementedtanks (n = 9)	**7.6±0.24**	**116.01± 23.05**	**0.21± 0.041**
Plasticbuckets (n = 3)	**6.9±0.82**	**103.33±17.52**	**0.19±0.032**
Plastic tanks (n = 4)	**7.4±0.58**	**105.86±35.9**	**0.19±0.065**
Earthy pots (n = 5)	**7.6±0.28**	**117.46±56.01**	**0.21±0.101**
Metal drum (n = 1)	**8.0±0.00**	**140.65±0.00**	**0.25±0.00**

## Discussion

Total 51(19.31%) serum samples out of 264 samples were positive for anti-dengue IgM antibody which is in agreement of the findings by Gaire et al [14]. The positivity for anti-dengue IgM reported by Sah et al was 30% [18] and that reported by Gupta et al was 29.09% [12]. Similarly, Poudel et al [19] and Shah et al [20] reported the positivity for anti-dengue IgM to be 12.17% and 8.99%, respectively. The reason for difference in positivity may be due to variation in the geography and effectiveness of the vector control programs in the epidemic regions as well as the demographic and social changes, urbanization and environmental changes.

The ratio of dengue seropositive male to female was 1:1.62 which supports the result of Gaire et al [14]. But more male were found to be affected in comparison to female by Poudel et al [19] and Gupta et al [12]. Statistically, there was no significant difference between genders and positive serological results.

There was significant difference in anti-dengue IgM seropositivity in the patients from hospital in Chitwan and those from hospitals in Dang (p<0.05). Higher numbers of positive cases from Chitwan might be due to the endemicity of dengue with many dengue outbreaks reported in this area [12].

Among the dengue seropositive cases, the common clinical features were fever, anorexia, headache, myalgia, nausea, retro-orbital pain, abdominal pain and skin rashes but no signs of hemorrhage were seen. The severity of these clinical symptoms is different in each patient depending on the immune system, infection with serotypes and multiple serotypes.

Thrombocytopenia (p<0.05) and leucopenia (p<0.05) were found significant whereas increased hematocrit level was not found significant in dengue seropositive cases. Thrombocytopenia and leucopenia are common in dengue in both mild and severe conditions [21]. In dengue fever the thrombocytopenia may be due to the destruction of the peripheral platelets or the destruction of the hematopoietic progenitor or bone marrow stromal cells by the virus, resulting in reduced production of platelets. Similarly, leucopenia may occur because of the virus-induced destruction or inhibition of myeloid progenitor cells [22]. In this study, BPR of the dengue vectors (*Aedes spp*) was calculated to estimate the degree of breeding preference of dengue vectors toward particular container types. Eight different containers were searched for the immature dengue vectors. Discarded tires were found with the highest BPR of 1.15 and 1.14 in both Chitwan and Dang respectively, and was statistically significant (p<0.05). This revealed that discarded tires are the excellent breeding sites for dengue vectors. Similar findings were also found in the previous studies carried out in Nepal [14], India [23] and Philipines [24]. The reason for highest breeding preference of dengue vectors in the discarded tires may be due to the fact that tires are discarded near the houses and remain undisturbed for long period of time. Tires are less susceptible to water loss because of the shape as well as they shield the water surface from wind and sun, resulting in slower evaporation rate [14].

The article "Serological and Entomological Study of Dengue in Dang and Chitwan Districts of Nepal" was retracted in 2022. Reason: lack of ethics approval or compliance.

Different entomological indices were used for the study of distribution and density of dengue vectors in the study areas. BI in Chitwan was found to be significantly higher in comparison to that in Dang (p<0.05). Statistically, there was no significant difference between AI and CI of Chitwan and those of Dang. The serological study of the Chitwan and Dang showed that the numbers of seropositive cases (37.6%) were higher in Chitwan where the BI was found higher. In case of Dang, the sero-positive (2.88%) cases were found lower than Chitwan. This suggests that sero-positivity increases with increase in the BI and this entomological index may be useful in determining the higher risk geographical areas for dengue and early warning for dengue outbreak.

The physiochemical characteristics of water of the habitats of *Aedes* mosquito were determined. The physiochemical parameters are the important abiotic factors for the survival and development of the mosquito larva. In this study, pH, chloride ions concentration and salinity of the water collected from different types of the containers were determined. Similar study done by Umar and Don-Pedro [25], showed that the mosquitoes prefer the breeding habitat with the pH ranging from 6.5 to 8 whereas the study done by Clarket al [26] and Glenn et al [27], showed that mosquitoes prefer to breed in habitats with pH ranging from 4 to 11 and 4 to 9 respectively.

The article "Serological and Entomological Study of Dengue in Dang and Chitwan Districts of Nepal" was retracted in 2022. Reason: lack of ethics approval or compliance.

The rise in the salinity of the mosquito habitats could be an indicator for the emergence of salinity tolerant mosquitoes. These physiochemical parameters are important to know the conditions required for the oviposition of the mosquitoes as well as for the development and survival of the mosquito’s larva. Previous study done by Bradley, [28] and Nguyan and Donine, [29] indicated that although salinity is the important parameter for the development of the mosquito different mosquitoes would have specific tolerance that enable them to osmo-regulate and adapt to varying salinity in the water.

## Conclusion

Fifty one (19.31%) out of 264 samples were found positive for anti-dengue IgM antibody by capture ELISA. This study is an attempt to highlight the relationship between the hematological features (leukocytes count and thrombocytes count) and clinical features with dengue virus infection, which would be useful for the suspection of the disease in its early stage and hence to diagnose it immediately. The decreased thrombocytes count and leucocytes count along with clinical symptoms like fever, anorexia, nausea, myalgia, headache, retro-orbital pain and skin rash might be suggestive for dengue virus infection.

The determination of BPR revealed that discarded tires are the excellent breeding habitat for the vector and BI was found higher in Chitwan than that in Dang district. Different physiochemical analysis of the breeding habitats showed that the breeding water of *Aedes* mosquito had wide range of pH ranging from slightly acidic to basic with chloride ion concentration ranging from 140.65 mg/L to 103.33 ± 17.52 mg/L and salinity ranging from 0.25ppt to 0.19±0.032 ppt. The proper vector management programs and environmental education strategies along with knowledge about physiochemical properties of the breeding habitats of *Aedes* are essential for reducing the vectors and hence to control the dengue.

## Supporting Information

S1 File Hematological features of the anti-dengue IgM seropositive cases. (DOCX)

S2 File Raw data for leucocyte count, thrombocyte count and hematocrit level of the anti-dengue IgM seropositive cases. (SAV)
